# Metabolomic Identification of Serum Exosome-Derived Biomarkers for Bipolar Disorder

**DOI:** 10.1155/2022/5717445

**Published:** 2022-01-10

**Authors:** Yang Du, Ji-Hui Dong, Lei Chen, Hua Liu, Guang-En Zheng, Guang-Yang Chen, Yong Cheng

**Affiliations:** ^1^Key Laboratory of Ethnomedicine of Ministry of Education, Center on Translational Neuroscience, School of Pharmacy, Minzu University of China, Beijing, China; ^2^The Third People's Hospital of Foshan, Foshan, Guangdong, China; ^3^NHC Key Laboratory of Birth Defects Research, Prevention, and Treatment, Hunan Provincial Maternal and Child Health-Care Hospital, Changsha, Hunan, China

## Abstract

**Background:**

Exosomes are extracellular vesicles that play important roles in various physiological and pathological functions. Previous studies have demonstrated that exosome-derived contents are promising biomarkers to inform the pathogenesis and diagnosis of major depressive disorder and schizophrenia.

**Methods:**

We used ultraperformance liquid chromatography-tandem mass spectrometry to analyze the differentially expressed metabolites in serum exosomes of patients with bipolar disorder (BD) and evaluated the potential of exosomal metabolites as biomarkers for BD.

**Results:**

Our results showed 26 differentially expressed serum exosomal metabolites in patients with BD (*n* = 32) when compared with healthy control (HC) subjects (*n* = 40), and these differentially expressed metabolites were enriched in pathways related to sugar metabolism. We then utilized random forest classifier and identified 15 exosomal metabolites that can be used to classify samples from patients with BD and HC subjects with 0.838 accuracy (95% CI, 0.604–1.00) in the training set of participants. These 15 metabolites showed excellent performance in differentiating between patients with BD and HC subjects in the testing set of participants, with 0.971 accuracy (95% CI, 0.865–1.00). Importantly, the 15 exosomal metabolites also showed good to excellent performance in differentiating between BD patients and other major psychiatric diseases (major depressive disorder and schizophrenia).

**Conclusion:**

Collectively, our findings for the first time revealed a potential role of exosomal metabolite dysregulations in the onset and/or development of BD and suggested that blood exosomal metabolites are strong candidates to inform the diagnosis of BD.

## 1. Introduction

Bipolar disorder (BD) is a common and debilitating neuropsychiatric disorder that may cause functional impairments, important disabilities, and premature death with huge burden for society and affected families and individuals [1, 2]. BD is generally considered to be caused by the complex interaction between genetic and environmental factors, although the molecular mechanism underlying the pathogenesis of the disease is still poorly understood [3]. The disease comprises periods of depression, mania, and euthymia, and the diagnosis is made based on solely subjective evaluations of clinicians, without objective methods, which may result in a considerable error rate [4]. Over the last two decades, great efforts have been made to identify biomarkers for BD diagnosis and treatment response, and to assist the elucidation of the etiology of the devastating disease.

In recent years, the field has grown to encompass multiomic techniques to biomarker discovery in mental disorders, including major depressive disorder (MDD), schizophrenia (SCZ), and BD. A substantial number of studies have utilized proteomics, metabolomics, and RNA sequencing and discovered potential biomarkers to support the diagnosis of these major neuropsychiatric diseases [5, 6]. Of particularly interesting is that a number of studies have found potential biomarkers from blood exosomes to inform the diagnosis and/or treatment response of MDD and SCZ [7–11]. Given that exosomes can cross blood-brain barrier easily, and therefore, the changes of blood exosomal contents in patients with neuropsychiatric diseases were hypothesized to be at least partially reflect central changes [8], Wei et al. utilized a genome-wide miRNA expression profiling of blood-derived exosomes from patients with MDD and healthy control (HC) subjects and found a set of miRNAs were able to differentiate between MDD patients and controls, suggesting the potential of exosome-derived miRNAs as diagnostic markers for MDD. These miRNAs included miR-139-5p, which was shown as a negative regulator for neural stem cell proliferation and neuronal differentiation, and thereby modulating depressive-like behaviors in mice [11]. Additionally, our group found 11 miRNAs in blood exosomes from the miRNA sequence data had good performance to distinguish between SCZ patients and controls and also suggested that medications differentially regulated the miRNA levels in SCZ patients [8]. We subsequently performed a multicenter study and revealed that a set of metabolites from blood exosomes had strong potential to inform the diagnosis of SCZ. Bioinformatics analysis indicated that the differentially expressed blood exosomal miRNAs or metabolites were involved in the pathophysiology of SCZ [7]. These results indicated that biomarkers from blood exosomes are good candidates for objective diagnosis of major psychiatric diseases and also have potentials to elucidate the molecular mechanisms underlying the pathogenesis of these diseases. However, the potential role of blood exosome-derived contents in the etiology and diagnosis of BD is unclear.

Here, we performed the first ultraperformance liquid chromatography–tandem mass spectrometry (UPLC-MS/MS) study to analyze the blood exosome metabolomic profile of BD patients and HC subjects. We found a set of differentially expressed exosomal metabolites in patients with BD, which were enriched in pathways related to sugar metabolism. Additionally, we identified 15 metabolites as promising biomarkers to inform the diagnosis of BD.

## 2. Materials and Methods

### 2.1. Participants

BD (*n* = 32), SCZ (*n* = 42), and MDD (*n* = 31) patients and HCs (*n* = 40) were recruited from the Third People's Hospital of Foshan, Foshan, Guangdong, China. The diagnosis of BD and MDD patients were made by experienced psychiatrists according to The International Classification of Diseases-10 and The Structured Clinical Interview of DSM-5. The patients' psychiatric symptoms were assessed by Hamilton Depression Scale (HAMD) and Bech-Rafaelsdn Mania Rating Scale (BRMS). Any individuals with physical or medical illness were excluded from this study. The demographic and clinical characteristics of the BD patients and HC subjects are presented in Table 1.

All the participants signed a written informed consent. The study protocol was reviewed and approved by the biological and medical ethics committee, Minzu University of China. The experiments were conducted in accordance with the Declaration of Helsinki.

### 2.2. Exosome Isolation and Validation

The exosome isolation and validation were performed as described in our previous paper [7]. Briefly, the serum samples from patients and controls were collected, and serum exosomes were obtained on a qEV column. The exosome validation methods negative-staining electron microscopy, nanoparticle tracking analysis, and Western blotting were also presented in our recently published paper [8].

### 2.3. Metabolite Measurements

The serum exosome samples from patients and controls were subjected to widely targeted metabolomics analysis through an UPLC-MS/MS as described previously [7]. Briefly, the public database of metabolite information and metabolomics data curation environment (MetWare) was performed to achieve qualitative analysis of the first- and second-order mass spectra. The quantification of metabolites was achieved through multiple reaction monitoring and triple quadrupole mass spectrometry.

### 2.4. Random Forest Classifier

A 10-fold crossvalidation was performed on a random forest model (R 3.2.4, randomForest package) using the metabolite abundance profile of the BD patient samples and control samples. The crossvalidation error curves (average of 10 test sets each) from 5 trials of the 10-fold crossvalidation were averaged, and the minimum error in the averaged curve plus the standard deviation (s.d.) at that point was used as the cutoff. All sets of metabolite markers with an error less than the cutoff were listed, and the set with the smallest number of metabolite markers was chosen as the optimal set. A receiver-operating characteristic (ROC) was drawn (R 3.2.4, pROC package) to assess the accuracy of this set of metabolite markers to diagnose BD. To validate the potential of the biomarkers to diagnose BD, the model was further tested on a testing set.

### 2.5. Weighted Gene Coexpression Network Analysis

Coexpression network analysis was performed by the WGCNA R package which has been employed in metabolite coexpression study [12]. The Pearson's correlation was used to assess correlations between metabolites, and the soft-thresholding power was chosen based on the criterion of approximate scale-free topology. A signed coexpression network was then constructed by assigning metabolites to modules using cutreeDynamic function. For module-trait analyses, the Pearson's correlation was calculated between module expression (defined as the first principle component of all metabolites in a module) and diagnosis status, age, gender, and disease severity. The potential hub nodes or metabolites within each module with high intramodular importance were also identified. Significant module-trait results were reported at Benjamini-Hochberg corrected *p* < 0.05.

### 2.6. Kyoto Encyclopedia of Genes and Genomes (KEGG) Database

To systematically elucidate the potential biological functions of the differentially expressed metabolites and hub metabolites in a module, these metabolites were subjected to the KEGG pathway database analysis by the MetaboAnalyst software [13]. We defined significant enrichment pathways as *p* < 0.05.

### 2.7. Statistical Analysis

We applied principal components analysis (PCA) to identify outliers. Differentially expressed metabolites were identified through partial least squares discriminant analysis (OPLS-DA) model, which was used to extract the variable importance in projection (VIP) [14]. Differentially expressed metabolites were defined as VIP > 1.0. These analyses were performed by SIMCA software (version 14.1). Additionally, the ROC curves generated by the SPSS 22.0 statistical analysis software [15] were used to assess the potential of serum exosomal metabolites as biomarkers to distinguish BD patients from disease controls.

## 3. Results

### 3.1. Differential Expression of Serum Exosomal Metabolites in BD

Metabolomic profiling detected 350 compounds (samples from BD patients and controls) which passed quality control procedures and were eligible for analysis. Plots of PCA scores showed a separation of metabolite profiles between BD patients and controls (Figure 1(a)), suggesting the presence of a BD signature in the blood exosomal metabolite concentrations. To identify differentially expressed blood exosomal metabolites between BD patients and controls, an OPLS-DA model was constructed (Figure 1(b)), which identified 26 metabolites by the criteria: VIP score > 1.0 (Figures 1(c) and 1(d)). Of these, 11 were upregulated and 15 were downregulated (Figures 1(c) and 1(d)). Significant KEGG pathway enrichment was found for the differentially expressed metabolites in pathways related to galactose metabolism and amino sugar and nucleotide sugar metabolism (Figure 1(e)).

### 3.2. Exosomal Metabolites as Biomarkers for BD

Given the robust associations of some exosomal metabolites with BD, we therefore explored whether exosomal metabolites could be served as biomarkers to differentiate between BD patients and HC subjects. A total of 350 metabolites from the training set of participants were subjected to random forest classifier for potential metabolite biomarker analyses, and a set of 15 metabolites (Chenodeoxycholic Acid, Lysope 18 : 0, Lysope 14 : 0, N-Acetylmethionine, 13-oxoODE, Glycine, 1-Naphthylacetic Acid, 2-Aminoethanesulfonic Acid, D-2-Aminobutyric Acid, Lysopc 18 : 0, Lysopc 20 : 1, Biopterin, Phosphoric Acid, and Glucosamine, PAF C-16) were identified as the optimal set of metabolites to discriminate between BD patients and HC subjects. We used the 15 metabolites to draw a ROC curve in the training set of participants, and the area under curve (AUC) was 0.838 (95% CI, 0.604–1.00) (Figure 2(a)). We next applied the 15 metabolites to the testing set of participants for class prediction, and the AUC was 0.971 (95% CI, 0.865–1.00; Figure 2(b)). These results suggested that the 15 blood exosomal metabolites may be biomarkers to inform the diagnosis of BD.

To investigate whether these potential biomarkers were specific to BD, we used the 15 metabolites to draw ROC curves to test whether they can distinguish BD patients from other major neuropsychiatric diseases, such SCZ and MDD. The ROC curve included 42 patients with SCZ and 32 patients with BD, and yielded an AUC of 0.886 (95%CI = 0.774–0.972) to discriminate between BD patients and SCZ patients (Figure 3(a)). Another ROC curve included 31 patients with MDD and 32 patients with BD, and yielded an AUC was 0.771 (95%CI = 0.614–0.940) to discriminate between BD patients and MDD patients (Figure 3(b)). These results demonstrated that blood exosomal metabolites are strong candidates to inform the diagnosis of BD.

### 3.3. Perturbation of Exosomal Metabolite Coexpression Modules in BD

To better understand the relationship between blood exosomal metabolite changes and disease status at a systems level, 72 samples (32 BD patients and 40 HC subjects) were subjected to WGCNA to assign individual metabolites to coexpression modules, which resulted in the identification of 4 modules (Figure 4(a)). We then calculated correlation between the first principal component of each module and disease status and identified turquoise and blue modules that were significantly correlated with disease status (Figure 4(b)). Additionally, turquoise module was significantly associated with BRMS, and blue module showed significant associations with age and HAMD (Figure 4(b)), suggesting the potential confounding effects of clinical variables on the blood exosomal metabolite levels. Besides, we identified 20 potential hub nodes or metabolites within blue (Figure 4(c)) and turquoise (Figure 4(d)) modules with high intramodular importance. KEGG pathway analyses indicated that the top three significantly enriched pathways in blue module are valine, leucine, and isoleucine biosynthesis, aminoacyl-tRNA biosynthesis, and phenylalanine, tyrosine, and tryptophan biosynthesis pathway (Figure 4(e)).

## 4. Discussion

Our metabolomics data demonstrated 26 differentially expressed metabolites in the blood exosomes of patients with BD relative to HC subjects. Bioinformatics analysis identified 15 metabolites in the blood exosomes which had good to excellent performance in distinguishing between BD patients and HC subjects. The potential of the 15 metabolites to discriminate between BD patients and controls was validated by a testing set of participants in the same clinical center, suggesting the robustness of the data that these metabolites from blood exosomes can distinguish BD patients from HC subjects. Additionally, the 15 metabolites showed good to excellent performance in discriminating between BD patients and other major neuropsychiatric diseases (MDD and SCZ), indicating that these exosomal metabolites are promising biomarkers to diagnose BD in practice in the future. Further WGCNA analysis showed four coexpression modules from 72 samples (32 BD patients and 40 HC subjects), and several modules were associated with age, diagnosis, and severity, suggesting that age and disease severity were potential confounders for blood exosomal metabolite levels in BD patients. Taken together, we provided first evidence of blood exosomal metabolite dysregulation in patients with BD and also provided new perspectives into the roles of metabolites in BD diagnosis and pathophysiology.

Our bioinformatics analysis revealed the top three enrichment pathways for the differentially expressed blood exosomal metabolites were galactose metabolism, amino sugar and nucleotide sugar metabolism, and pentose and glucuronate interconversions, suggesting a potential role of sugar metabolism dysfunction in the onset and/or development of BP. The role of sugar metabolism in the BP pathogenesis was supported by the data from Wei et al.; they recruited 91 patients with bipolar disorder and 92 HC subjects and found amino sugar metabolism was altered in plasma of patients with bipolar disorder compared to HC subjects [16]. Additionally, a postmortem study showed that several sugar metabolites in the brains of the patients were different between BP patients and control subjects; these metabolites included sorbitol, gluconic acid, and erythritol as determined by LC-MS analysis [17]. These above results all showed sugar metabolism imbalance in patients with BP which may provide novel and critical information to support the elucidation and/or new insights into the molecular pathways underlying BP pathogenesis and also provides a potential therapeutic target for the treatment of BP.

Over the last two decades, growing number of studies tried to search biomarkers from blood for BD, partly due to the “peripheral as a window on the brain” hypothesis [18], and blood samples are easily accessible. These efforts have led to discovery of potential biomarkers for BD, including miRNAs, neurotrophic factors, and metabolites [1, 19]. Interestingly, a dysregulation of the kynurenine pathway has been observed in patients with BD, and this was summarized by a recent meta-analysis, which showed lower peripheral blood tryptophan, kynurenine, kynurenic acid, and xanthurenic acid levels in BD patients than that of HC subjects [20], suggesting the potential of these metabolites as biomarkers for BD. However, these studies have not translated into clinical practice. One problem is the specificity for the potential biomarkers to differentiate between BD patients and other psychiatric patients, although a recent study employed proton magnetic resonance spectroscopy and provided potential peripheral blood metabolite biomarkers to allow differential diagnosis between BD and SCZ [21]. Here, we uncovered a set of metabolites from serum exosomes and not only differentiate between BD patients and HC subjects but also discriminate between BD patients and disease controls (patients with MDD and SCZ), indicating the strong potential of these metabolites to inform the diagnosis of BD. Therefore, future studies are necessary to validate the potential of blood exosome-derived metabolites as diagnostic biomarkers for BD.

Notably, the potential metabolite biomarkers included many lipids, especially phospholipids, such as lysoPE 18 : 0, lysoPE 14 : 0, lysoPC 18 : 0, and lysoPC 20 : 1. Previous studies have shown evidence for alterations in phospholipids and their fatty acids in patients with BD. For example, arachadonic and docosahexaenoic acid were found to be reduced in red blood cell membranes of BD patients in a manic phase [22]. Another study used *in vivo* proton magnetic resonance spectroscopy and found increased glycerophosphocholine plus phosphocholine levels in the basal ganglia and anterior cingulate cortex of patients with BD, which are brain regions that are important for mood regulation [23]. Moreover, Knowles et al. recruited a sample of 558 individuals from 38 extended pedigrees and analyzed 13 serum-based phospholipid concentrations; they concluded that serum-based phosphatidylinositol had a significant association with BD risk [24]. Additionally, the potential biomarkers included 13-oxoODE, which belongs to oxidized linoleic acid metabolites, and have been implicated in various pathological conditions [25]. These results suggested oxidative stress may be implicated in the blood exosomal metabolite dysfunction leading to the pathogenesis. Data from the two previous studies supported this hypothesis, as lipid peroxidation levels in plasma have been shown to be increased in euthymic adults with BD [26]. In contrast, lipid peroxidation levels were found to be decreased in adolescent BD patients [27]. These results all suggested a critical role of the membrane phospholipid and oxidative stress in the onset and/or development of BD, although between-study heterogeneities were observed on metabolite levels in BD patients, which may be confounded by population, testing methodology, disease severity, and disease stage. Additionally, a limitation of this study is that the sample size is relatively small, which requires future studies with large sample size to validate the data from the present study. Another limitation is that absolute quantification of the potential BD biomarkers was not achieved in this study. Therefore, further investigations are warranted to analyze these metabolites from blood exosomes, hopefully with international cooperation, to result in breakthroughs on blood biomarkers capable of informing BD diagnosis.

## Figures and Tables

**Figure 1:** Identification of differentially expressed serum exosomal metabolites in bipolar disorder (BD). (a) Principal components analysis (PCA) and (b) an orthogonal partial least squares discriminant analysis (OPLS-DA) model diagram according to the blood exosomal metabolites in the BD patients and healthy control (HC) subjects. (c) Heatmaps showing differentially expressed blood exosomal metabolites in patients with BD as compared to HC subjects. (d) Illustration of the 26 differentially expressed metabolites in BD. (e) KEGG enrichment pathways for the 26 serum exosomal metabolites differentially expressed in BD.

**Figure 2:** Biomarker performance for the set of 15 metabolites to discriminate BD patients from HC subjects. Receiver-operating characteristic (ROC) curves showing the accuracy of the 15 serum exosomal metabolites in distinguishing between BD patients and HC subjects in (a) the training participant set and (b) the test participant set.

**Figure 3:** Biomarker performance for the set of 15 metabolites to discriminate BD patients from disease controls. ROC curves showing the accuracy of the 15 serum exosomal metabolites in distinguishing between (a) BD patients and schizophrenia (SCZ) patients and (b) BD patients and major depressive disorder (MDD) patients.

**Figure 4:** Dysregulated serum exosomal metabolite coexpression modules in patients with BD. (a) Dendrogram showing metabolite coexpression modules defined in 72 samples (32 BD patients and 40 HC subjects). (b) Pearson's correlation coefficient between gender, age, disease status, disease severity, and module eigengene. (c, d) Coexpression hub node (metabolite) network plots for blue and turquoise modules. (e) KEGG enrichment pathways for the 20 hub nodes (metabolites) in blue and turquoise modules.

**Table 1:** Demographic and clinical characteristics of the study subjects.

Group		HC	BD
Training set	*N*	16	12
	Gender (male %)	37.5	33.3
	Age	25.5 ± 4.44	25.08 ± 5.55
	HAMD	\	10.08 ± 11.37
	BRMS	\	29.9 ± 7.80
Testing set	*N*	24	20
	Gender (male %)	29.1	25
	Age	22.5 ± 4.00	32.2 ± 8.48
	HAMD	\	10.6 ± 11.34
	BRMS	\	28.6 ± 10.02

Note: BD: bipolar disorder; HC: healthy control; HAMD: Hamilton Depression Scale; BRMS: Bech-Rafaelsen Mania Rating Scale.

## Data Availability

Data are available upon request.
